# Targeting Inhibition of Notch1 Signaling Pathway on the Study of Human Gastric Cancer Stem Cells with Chemosensitization

**DOI:** 10.1155/2022/1098394

**Published:** 2022-04-26

**Authors:** Yan Dou, Jinghong Wang

**Affiliations:** Clinical Laboratory, Huaihe Hospital of Henan University, Kaifeng 475000, Henan, China

## Abstract

**Background:**

Gastric cancer is the second most frequent cause of cancer death worldwide, although much geographical variation in incidence exists. Prevention and personalized treatment are regarded as the best options to reduce gastric cancer mortality rates (Hartgrink et al., 2009). Numerous studies have suggested that Notch1 and its ligands are overexpressed in gastric cancer, and its knockdown can inhibit the proliferation and survival of gastric cancer cells.

**Objective:**

To investigate the effect of Notch1 on the stemness and drug sensitivity of human gastric cancer SGC-7901 cells.

**Methods:**

Highly expressed Notch1 intracellular domain (NICD1) and Notch1-shRNA lentiviral expression vector were used to infect human gastric cancer SGC-7901 cells cultured in vitro, and western blot and immunofluorescence staining were used to identify highly expressed NICD and Notch1 silenced cells. The percentage of CD133+ cells was analyzed by flow cytometry, the expression of nestin and CFAP by immunofluorescence staining, the formation rate of tumor cell spheres and the tumorigenicity of SCID mice in vivo, and the regulation of cell stemness by Notch1. The sensitivity of each group of cells to the chemotherapeutic drugs teniposide (VM-26) and carmustine (BCNU) was also detected by the MTT method.

**Results:**

The stemness phenotype of tumor cells with the increased NICD expression was enhanced, such as an increased proportion of CD133+ cells, enhanced nestin expression, decreased GFAP expression, increased tumor cell sphere formation rate and tumorigenic rate of SCID mice implantation, and decreased sensitivity to VM-26 and BCNU. In contrast, the stemness phenotype of tumor cells with downregulated Notch1 gene expression was significantly suppressed, while the sensitivity to VM-26 and BCNU was increased.

**Conclusion:**

High Notch1 expression increased the stemness of SGC-7901 cells and decreased the sensitivity of SGC-7901 cells to chemotherapeutic drugs.

## 1. Introduction

Gastric cancer is the most common malignant tumor of the digestive system, and it is the second most frequent cause of cancer death worldwide, although much geographical variation in incidence exists. Surgery combined with chemotherapy is an important tool in the treatment of gastric cancer [1]. At present, the prognosis of conventional treatment for this tumor is still unsatisfactory, and one of the important factors for the poor effect of chemotherapy is the gradual development of secondary drug resistance in some of the tumor cells remaining after chemotherapy, which leads to the failure of chemotherapy and tumor recurrence [2,3]. The higher the proportion of CSCs in gastric cancer, the stronger the resistance of gastric cancer to chemotherapy [4,5]. The Notch signaling pathway is involved in regulating stem cell structure and determining cell fate. It has been shown that the Notch signaling pathway is associated with gastric carcinogenesis and development, and the Notch signaling was found to be overexpressed in gastric cancer, which plays an important role in the proliferation and differentiation of gastric cancer cells as well as apoptosis [6,7]. Farnie and Clarke [8] demonstrated evidence that upregulation of Notch expression is associated with breast cancer stem cells, suggesting that Notch and breast cancer stem cell-like features are related. A study by Zhang et al. [9] found that NICD, an activated form of Notch1, was detectable in SHG-44 and U87 cell lines. And these two gastric cancer cell lines proliferated faster than gastric cancer cell lines without detectable NICD. Numerous studies have suggested that Notch1 and its ligands are overexpressed in gastric cancer, and its knockdown can inhibit the proliferation and survival of gastric cancer cells. In gastric cancer, which is very closely related to Notch1, is Notch1 also an important factor in the development of stem cell-like phenotype in tumor cells [10–12]? Does it affect the sensitivity of cells to chemotherapeutic drugs? In this study, we investigated the regulation of Notch1 expression on the stem cell-like characteristics and sensitivity to chemotherapeutic drugs VM-26 and BCNU in gastric cancer SGC-7901 cells by transgenic regulation of Notch1 signaling, and the results showed that when Notch1 signaling was enhanced, SGC-7901 cells showed stronger characteristics of tumor stem cells, such as CD133+ tumor cells.

## 2. Materials and Methods

### 2.1. Experimental Materials

The Notch1 intracellular domain (NICD) expression vector pLVX-IRES2-ZsGreen-NICD was constructed and characterized by our laboratory and is referred to as pLVX-NICD. The empty control vector is called pLVX. The three plasmids lentiviral expression system carrying ZsGreen and the Notch1 gene RNA interference vector were kindly provided by Dr. Guo Ya from Shanghai Jiao Tong University. pLKO.1-puro interferes with the target sequence 5′-CCGGGACATCACGGATCATAT-3′ (referred to as pLKO-Notch1-ND). SCID mice were purchased from Shanghai Slaughter Experimental Animal Company, Certificate of Conformity No. 2007000579362, 2007000574540.2007000574540.

bFGF was purchased from Pep-roTech. Liposome Lipofectamine 2000 and MTT were purchased from Invitrogen. Rabbit anti-human NICD polyclonal antibody, rabbit anti-glial fibrillary acidic protein (GFAP) polyclonal antibody, rhodamine-labeled anti-rabbit IgG antibody, and rhodamine-labeled anti-mouse IgG antibody were purchased from Millipore. Mouse anti-CD133/1 (AC133)-PE antibody was purchased from Miltenyi Biotec. Mouse anti-nestin monoclonal antibody was purchased from R&D. Rabbit anti-GAPDH polyclonal antibody was purchased from Santa Cruz. HRP-coupled anti-rabbit IgG antibody and HRP-coupled anti-mouse IgG antibody were purchased from Beijing Zhongsun Jinqiao. Plasmid extraction and purification kit was purchased from QIAGEN. ECL chemiluminescence kit was purchased from CST. Carmustine (1,3-bis(2-chloroethyl)- 1-nitrosourea, 1, 3-bis (2-chloroethyl)-1 -nitrosourea; BCNU) and teniposide (VM-26) were purchased from Enzo Life Science. Puromycin was purchased from Amresco. Other reagents were purchased from Sigma or Beyoncé.

### 2.2. Acquisition of SGC-7901 Cells with High NICD Expression and Notch1 Knockdown SGC-7901 Cells

The pLVX-NICD, pLVX, pLKO- Notch1-ND, pLKO- Notch1-NC plasmids, and packaging plasmids pMD2.G and psPAX2 were obtained according to the conventional method in our laboratory. G and Lipofectamine 2000, respectively, and transfected 293T cells for viral packaging. The virus-containing culture supernatants were collected and concentrated at 48∼72 h of transfection. Gastric cancer cells SGC-7901 were routinely cultured in DMEM medium containing 10% fetal bovine serum and digested with 0.25% trypsin +0.03% EDTA once every 2∼3 d. The cells were inoculated in 6-well plates 1 d before infection, about ^5×104^ cells per well, and on the second day when about 30% fusion occurred, the culture medium was removed, and 600 *μ*L of serum-containing culture medium, 10 *μ*L of lentivirus solution, and 4.8 *μ*L of polybreen (1 g/L) were added to each well. 10 *μ*L, polybreen (1 g/L) 4.8 *μ*L, and incubated in the incubator for 12 h. After 12 h, the virus-containing culture medium was aspirated and replaced with 2 mL of fresh culture medium and incubated for 48 h at 37°C, 5% CO_2_, and saturated humidity. SGC-7901 cells with high NICD expression and their corresponding control cells were infected with the virus for 48 h. Notch1 gene RNA-interfering cells and their corresponding control cells were screened for successful infection with puromycin.

### 2.3. Identification of Notch1 Expression Level Western Blot Assay

Total cellular protein was extracted with RIPA cell lysate and protein concentration was determined by BCA method. After 40 *μ*g of protein samples were transferred to membrane blotting after SDS-PAGE electrophoresis, and after overnight action at 4°C by the blocking solution, rabbit anti-human NICD antibody or GAPDH antibody was used to bind to the antigen on the membrane, and sheep anti-rabbit HRP-coupled II antibody was used to react with it. Then, ECL chemiluminescence reagent was added, and images were acquired under the gel imaging system (Bio-Rad). ImageJ 2x software was used to. The grayscale values of the protein bands were calculated using ImageJ 2x software, and the grayscale ratio of the target band/internal reference band was used as the relative expression of Notch1.

Immunofluorescence staining was performed as follows: cells were cultured in 12-well plates placed on coverslips, and cells in the logarithmic growth phase were inoculated by adjusting the density and incubated for 48 h. The culture fluid was aspirated, washed three times with prechilled PBS, fixed in 4% paraformaldehyde at room temperature for 30 min, washed with PBS, and treated with 0.1% Triton X-100 cell permeabilization for 30 min. The cells were immunofluorescently stained with the corresponding antibodies in the usual way for 30 min and then restained with DAPI (5 mg/L) for 10 min. The antifluorescence bursting solution was used to seal the slices, which were observed and photographed under a laser confocal microscope (Leica).

### 2.4. Detection and Comparison of Cell Stemness in Each Group

Detection of CD133+ cells in each group was as follows. The cells in each group were digested by trypsin and collected, and the cell concentration was counted and adjusted to 1 × 10^9^/L. A blank control group and an isotype control group were set up. The cells of each group were aspirated 100 *μ*L into 1.5 mL EP tubes, centrifuged at 300×g for 10 min, and resuspended with 100 *μ*L of prechilled PBA. 1 *μ*L of PE-labeled CD133 antibody was added to the experimental group; 1 *μ*L of PE-labeled isotype control antibody, to the isotype control group; 1 *μ*L of PBA, to the blank control group. They were mixed well and incubated for 1 h at 4 °C in a refrigerator, protected from light. The cells were washed with 1 mL of PBA and centrifuged at 300×g for 10 min, and the supernatant was completely discarded. 500 *μ*L of PBA was used to resuspend the cells in each group. We adapted flow cytometry for detection.

Detection and analysis of nestin and GFAP expression in each group of cells were as follows. Immunofluorescence staining was performed as previously described, and the cells were cultured in 12-well plates placed on coverslips for 48h. The cells were washed three times with prechilled PBS, fixed with 4% paraformaldehyde, washed with PBS, permeabilized with 0.1% Triton X-100 cells, immunofluorescence stained with anti-nestin and GFAP antibodies and the corresponding II antibodies, and then restained with DAPI. The cells were observed and photographed under a laser confocal microscope.

SCID mice subcutaneous implantation tumorigenic assay SCID mice were kept at constant temperature (25∼27°C), thermostat and SPF conditions. The cells of NICD high expression group and its control group in the logarithmic growth period were prepared into single-cell suspension with the cell number of 1×103, 1×105, or 5×105 per 0.2 mL. The mice were divided into six groups with five mice each, and the skin of the axilla of SCID mice was disinfected with iodophor, and 0.2 mL of cells was inoculated subcutaneously in the axilla area by aspiration with a sterile syringe (No. 6 needle) and continued to be reared. After a total of 10 weeks of observation, the rats were executed by cervical medullary dissection. The tumor was peeled out intact, the surface adipose tissue was removed and weighed, and the long and short diameters (mm) of the tumor were measured separately with vernier calipers, and the tumor volume was calculated according to the formula: volume (^mm3^) = 4/3 × *π* × (long diameter/2) × (short diameter/2)^2^.

The tumor cell formation rate of each group was determined by trypsin digestion. The cells were inoculated in 24-well plates at 1 mL per well, that is, 104 cells per well, and each group of cells were inoculated in three wells. After 10 d of culture, the number of tumor spheres larger than 75 *μ*m in diameter was counted under the microscope, and the tumor sphere formation rate (%) = the number of tumor spheres larger than 75 *μ*m in diameter in each well/total number of original inoculated cells in each well × 100%.

Detection of multidrug resistance in each group of cells by MTT was as follows. The cells were treated with 1.5 *μ*mol/L VM-26 and 150 *μ*mol/L BCNU, respectively, referring to other literature and the experience of our laboratory. Cells at logarithmic growth stage were inoculated in 96-well plates at 7,000 cells per well. They were incubated for 12 h at 37 °C with 5% CO_2_, and then, the drugs were added at the determined concentrations, and six replicate wells were made for each group of cells. After the cells were incubated for 48 baths, 20 *μ*L of 5 g/L MTT solution was added to each well, and the supernatant was carefully aspirated after 4 h. 150 *μ*L of DMSO was added to each well and shaken on a shaker for 10 min to dissolve the crystals. Cell survival rate (%) = (drug administration group − blank control group)/(negative control group - blank control group) × 100%.

### 2.5. Statistical Treatment

We used SPSS 20.0 software for statistical analysis. The measurement data were expressed as mean ± standard deviation (mean ± SD) after testing for normality and chi-square. The means between groups were analyzed by one-way ANOVA with multiple samples. SNK-q test was used for comparison between the two groups. The difference between the two groups was at *P* < 0.05 which is considered statistically significant.

## 3. Results

### 3.1. Obtained SGC-7901 Cells with High NICD Expression and Low Notch1 Knockdown

Four groups of cells were obtained according to the aforementioned transfection and screening methods: NICD-high expressing SGC-7901 cells (pLVX-NICD), high expressing control null cells (pLVX), Notch1 knockdown SGC-7901 cells (pLKO- Notch1-ND), and RNA interference control cells (pLKO- Notch1-NC). The results of Western blot and immunofluorescence staining showed that the expression of Notch1 in SGC-7901 cells with high NICD expression and low Notch1 knockdown caused significant changes (Figures 1 and 2).

### 3.2. Regulation of Notch1 Expression on the Stemness Phenotype of SGC-7901 Cells

#### 3.2.1. Notch1 Expression Affects the CD133+ Phenotype of SGC-7901 Cells

Flow cytometry results showed that the percentage of CD133+ cells in SGC-7901 cells with high NICD expression was significantly higher than that in the control group, while the percentage of CD133+ cells in SGC-7901 cells with Notch1 gene RNA interference was reduced compared with the control group. The percentage of CD133+ cells in SGC-7901 cells with Notch1 gene RNA interference was reduced compared with the control group, as shown in Figure 3.

#### 3.2.2. Notch1 Expression Affects the Expression of Nestin and GFAP in SGC-7901 Cells

The results of immunofluorescence intensity assay showed that the expression of nestin protein in NICD high expression cells was significantly stronger than that in its control group, while the expression of GFAP was significantly weaker. The expression of nestin in Notch1 RNA interference group cells was significantly weaker, while the expression of GFAP was significantly enhanced. In contrast, the expression of GFAP was significantly enhanced in the Notch1 gene RNA interference group, as shown in Figures 4 and 5 and Table 1.

#### 3.2.3. Notch1 Expression Affects the Tumor Sphere Formation Rate of SGC-7901 Cells

The tumor sphere formation rate of the NICD high expression group was significantly higher than that of its control group, which was 2.05 times higher than that of the control group. In contrast, the tumor sphere formation rate in the Notch1 gene RNA interference group was significantly lower than that in the control group, as shown in Figure 6.

#### 3.2.4. Increased Tumorigenic Ability of SGC-7901 Cells with High Expression of NICD in SCID Mice

The tumor size was 120.64 ± 42.51 mm3 and tumor weight was 0.21 ± 0.11 g, while only one of the five SCID mice in the control group had a tumor size of 78 mm3 and tumor weight of 0.10 g. See Figure 7.

### 3.3. Notch1 Expression Affects the Sensitivity of SGC-7901 Cells to Chemotherapeutic Drugs

The results of MTT method showed that the cell survival rate of NICD high expression group was significantly higher than its control group under the same concentration of VM-26 or BCNU, while the cell survival rate of Notch1 gene RNA interference group was significantly lower than that of the interference control group (Figure 8).

## 4. Discussions

Gastric cancer is the second most frequent cause of cancer death worldwide, although much geographical variation in incidence exists. Prevention and personalized treatment are regarded as the best options to reduce gastric cancer mortality rates [13]. Numerous studies have suggested that Notch1 and its ligands are overexpressed in gastric cancer, and its knockdown can inhibit the proliferation and survival of gastric cancer cells. It has been shown that the Notch signaling pathway is associated with gastric carcinogenesis and development, and the Notch signaling was overexpressed in gastric cancer, which plays an important role in the proliferation and differentiation of gastric cancer cells and apoptosis [6,7]. In this study, we investigated the regulation of Notch1 expression on the stem cell-like characteristics and sensitivity to chemotherapeutic drugs VM-26 and BCNU in gastric cancer SGC-7901 cells by transgenic regulation of Notch1 signaling. The results showed that when Notch1 signaling was enhanced, SGC-7901 cells showed stronger characteristics of tumor stem cells, such as CD133+ tumor cells The results showed that SGC-7901 cells showed stronger characteristics of tumor stem cells, such as more CD133+ tumor cells, increased nestin expression and decreased GFAP expression, increased tumor sphere formation, increased tumorigenicity of SCID mice subcutaneously transplanted, and significantly increased resistance to both VM-26 and BCNU when Notch1 signaling was enhanced. This suggests that the detection of Notch1 expression levels should be emphasized in gastric cancer research and treatment, and it is expected to be a potential target for regulating the sensitivity of gastric cancer chemotherapy.

At present, the prognosis of conventional treatment for this tumor is still unsatisfactory. The higher the proportion of CSCs in gastric cancer, the stronger the resistance of gastric cancer to chemotherapy [4, 5]. Notch signaling pathway is involved in regulating stem cell structure and determining cell fate. One of the important factors for the poor effect of chemotherapy is the gradual development of secondary drug resistance in some of the tumor cells remaining after chemotherapy, which leads to the failure of chemotherapy and tumor recurrence [2,3]. Overcoming the resistance of tumor cells to chemotherapeutic drugs is an important element in improving tumor outcomes, and the concept of CSCs has opened up a new space for the study of drug resistance in tumor cells, which is thought to play an important role in drug resistance and tumor metastasis because CSCs can express drug transport proteins and enhance DNA repair systems, thus making CSCs resistant to drugs. There is evidence that the Notch signaling pathway is associated with CSCs; for example, the pathway is involved in regulating stem cell populations in colorectal cancer [14] and also plays an important role in maintaining a CSCs-like phenotype in pancreatic cancer [15]. In this experiment, we further confirmed that high expression of Notch1 signaling could cause a stem cell-like phenotype of gastric cancer cells by transgenic overexpression of NICD.

Chemotherapy is an important treatment in cancer therapy. However, because of drug resistance, chemotherapy cannot destroy all tumor cells, which is the most important reason for tumor recurrence. Recently, a study reported that Notch signaling pathway is associated with drug resistance. More importantly, Notch regulates the formation of tumor stem cells and promotes the acquisition of epithelial-mesenchymal transition phenotype by cells, which is significantly associated with drug resistance [16]. Many studies have found that inhibition of Notch1 expression in many tumors, such as breast, pancreatic, and colon cancers, increases the sensitivity of tumor cells to chemotherapeutic drugs. Silencing Notch1 gene can activate p53 and promote PUMA and NOXA protein expression through activation of JNK1 signaling pathway, which in turn leads to apoptosis of human breast cancer MCF-7 cells through the mitochondrial pathway. Farnie et al. [8] demonstrated evidence that upregulation of Notch expression is associated with breast cancer stem cells, suggesting that Notch and breast cancer stem cell-like features are related. A study by Zhang et al. [9] found that NICD, an activated form of Notch1, was detectable in SHG-44 and U87 cell lines, and that these two gastric cancer cell lines proliferated faster than gastric cancer cell lines without detectable NICD; overexpression of NICD in SHG-44 cells promoted SHG-44 cell growth and colony formation; these colonies expressed nestin for cells with a neural stem cell phenotype. Hulleman et al. [6] found that the transcription factor HEY1, a downstream target molecule of the Notch signaling pathway, was significantly upregulated in gastric cancer and that HEY1 expression in glioblastoma multiforme correlated with tumor grade and survival, and that silencing HEY1 by RNA interference technology would cause glioblastoma in tissue culture to diminished proliferation. In gastric cancer stem cells, interferon regulatory factor 7 inhibits interleukin-6-Janus kinase signaling and Jagged-Notch signaling pathway activation, resulting in decreased expression of gastric cancer stem cell markers and reduced tumor cell sphere formation capacity and tumorigenicity [17]. In gastric cancer, inhibition of the Notch signaling pathway enhanced the sensitivity of CD133+ gastric cancer cells to the chemotherapeutic drug temozolomide. The results of this experiment also suggest that SGC-7901 cells exhibit stronger characteristics of tumor stem cells when Notch1 signaling is enhanced, and resistance to VM-26 and BCNU is also significantly enhanced. The most common causes of tumor drug resistance have been reported to be the expression of one or more energy-dependent transporter proteins (which detect chemotherapeutic drugs in cells and expel them), drug-induced apoptosis, and drug-induced detoxification malfunction. For example, ABC drug transporter proteins protect tumor cells from chemotherapeutic drugs. ABCC1 (multidrug resistance-associated protein 1; MRP1), ABCB1 (P-glycoprotein), and ABCG2 (breast cancer drug resistance protein), ABC transporter proteins, have been identified. MRP1 has been found to be associated with drug resistance in neurogastric carcinoma. MRP1 expression was detected in both neurogastric cancer tissues and gastric cancer cell lines. Calatozzolo et al. found a positive rate of 70% for MRP1 in human gastric cancer tissue sections, no significant grade variability in gastric cancer grades II, III, and IV, and no significant difference in primary and recurrent gastric cancer. Spiegl-Kreinecker et al. [22] showed that as the malignant grade of gastric cancer increased, MRP1 showed a gradual increase in positivity. High Notch1 expression increased the stemness of SGC-7901 cells and decreased the sensitivity of SGC-7901 cells to chemotherapeutic drugs.

## 5. Conclusion

The present experimental study showed that enhanced Notch1 signaling could promote the formation and proliferation of tumor stem cell-like cells and affect the sensitivity of neural gastric cancer cells to chemotherapeutic drugs. Therefore, Notch1 expression level can be used as an indicator to determine the stemness of gastric cancer and predict the sensitivity of chemotherapy, and the intervention of Notch1 signaling is expected to be an intervention target for gastric cancer treatment to overcome its drug resistance effect and kill gastric cancer stem cell-like cells to improve the chemotherapeutic effect on gastric cancer.

However, there are still limitations in this research. The relationship between Notch1 expression level and chemotherapy sensitivity is not clear, and we need further clinical trials. More experiments will establish the relationship between Notch1 and the sensitivity of chemotherapy and provide a more authoritative evaluation system for chemotherapy sensitivity.

## Figures and Tables

**Figure 1:** The protein expression of Notch1 in each group detected by western blot. Mean ± SD. *n* = 3. ^∗∗^*P* < 0.01 vs. pLVX; ^##^P < 0.01 vs pLKO-Notch1-NC the protein expression of Notch1 in each group was detected by western blot.

**Figure 2:** Identification of NICD expression in each group of cells by immunofluorescence staining.

**Figure 3:** Percentage of CD133 + cells in each group of cells. Mean ± SD. *n* = 3. ^∗∗^*P* < 0.01 vs. pLVX; ^##^*P* < 0.01 vs. pLKO-Notch1-NC.

**Figure 4:** The expression of nestin (red) in each group detected by immunofluorescence staining.

**Figure 5:** The expression of GFAP (red) in each group detected by immunofluorescence staining.

**Figure 6:** The formation rate of tumor spheres in each group cultured with stem cell medium. Mean ± SD. *n* = 3. ^*∗*^*P* < 0.05 vs. pLVX; ^#^P < 0.05 vs pLKO-Notch1-NC. The rate of formation of tumor spheres in each group cultured with stem cell medium.

**Figure 7:** Overexpression of NICD enhanced the formation of xenograft tumor in SCID mice.

**Figure 8:** The effects of chemotherapeutics on the survival rate of the cells with different treatments. Mean ± SD. *n* = 3. ^∗∗^*P* < 0.01 vs. pLVX; ^##^*P* < 0.01 vs. pLKO-Notch1-NC.

**Table 1:** The expression of nestin and GFAP in each group (mean ± SD; *n* = 3).

Group	Value of immunofluorescence	
	Nestin	GFAP
pLVX	36.23 ± 7.84	25.55 ± 3.73
pLVX-NICD	60.75 ± 11.98^∗∗^	12.06 ± 1.79^∗∗^
pLKO-Notch1-NC	34.40 ± 6.56	31.36 ± 5.64
pLKO-Notch1-ND	22.40± 6.48^##^	89.00 ± 15.28^##^

^∗∗^ *P* < 0.01 vs. pLVX; ^##^*P* < 0.01 vs. pLKO-Notch1-NC.

## Data Availability

The datasets used and/or analyzed during the current study are available from the corresponding author upon reasonable request.
